# A ceRNA Network Composed of Survival-Related lncRNAs, miRNAs, and mRNAs in Clear Cell Renal Carcinoma

**DOI:** 10.1155/2022/8504441

**Published:** 2022-04-28

**Authors:** Wenjun Lu, Hengchen Liu, Xin Zhang, Yujun Guo, Lu Liu, Tieyun Guo, Liqin Qu, Shulong Yang, Zhaozhu Li

**Affiliations:** ^1^Department of Pediatric Surgery, The Second Hospital Affiliated to Harbin Medical University, Harbin, Heilongjiang Province, China; ^2^Department of Basic Medicine College, Harbin Medical University, Harbin, Heilongjiang Province, China

## Abstract

Clear cell renal carcinoma (ccRCC) is one of the most common renal carcinomas worldwide, which has worse prognosis compared with other subtypes of tumors. We propose a potential RNA regulatory mechanism associated with ccRCC progression. Accordingly, we screened out clinical factors and the expression of RNAs and miRNAs of ccRCC from the TCGA database. 9 lncRNAs (FGF12-AS2, WT1-AS, TRIM36-IT1, AC009093.1, LINC00443, TCL6, COL18A1-AS1, AC110619.1, HOTTIP), 2 miRNAs (mir-155 and mir-21), and 3 mRNAs (COL4A4, ERMP1, PRELID2) were selected from differential expression RNAs and built predictive survival models. The survival models performed very well in predicting prognosis and were found to be highly correlated with tumor stage. In addition, the survival-related lncRNA-miRNA-mRNA (ceRNA) network was constructed by 18 RNAs including 12 mRNAs, 2 miRNAs, and 4 lncRNAs. It is found that the “ECM-receptor interaction,” “Pathways in cancer,” and “Chemokine signaling pathway” as the main pathways in KEGG pathway analysis. Overall, we established predictive survival model and ceRNA network based on multivariate Cox regression analysis. It may open a new approach and potential biomarkers for clinical prognosis and treatment of ccRCC patients.

## 1. Introduction

Clear cell renal carcinoma (ccRCC) is the most common pathological type of renal cancer (~80%); it has worse survival outcomes compared with other subtypes of tumors [1]. And its incidence rate has increased worldwide with each passing year. Therefore, investigated the underlying molecular mechanisms and the progression of ccRCC and new novel targets are urgently needed. The ceRNA network plays an important role in the field of tumor research [2]. ceRNA networks link the function of protein-coding mRNAs with that of noncoding RNAs such as microRNA, long noncoding RNA, and circular RNA.

However, the roles and functions of the survival-related lncRNA-miRNA-mRNA ceRNA network in clear cell renal carcinoma (ccRCC) are still unclear. Long noncoding RNAs (lncRNAs) has no function of encoding protein. It can also be used as biomarkers for the prognosis and diagnosis in tumors [3–5]. In recent studies, lncRNAs and ccRCC were confirmed to be closely related; the downregulation of HOTAIRM1 in ccRCC suggests that it may play a role in renal differentiation and inhibition of HIF1 dependent angiogenesis [6]. MicroRNAs (miRNAs) are members of noncoding RNAs [7]. MicroRNAs (miRNAs) play an important negative regulatory role in downstream genes, and miRNAs centered regulatory networks are involved in many biological processes [8–10]. For instance, microRNA-206 is closely related to the pathological stage and poor prognosis of patients with ccRCC, which may be achieved by targeted regulation of ZEB2 [11]. MicroRNA is a highly conserved endogenous noncoding RNA that interacts with target mRNA and downregulates its gene expression. In the process of gene expression, other RNA transcripts regulate biological processes by competing for shared miRNAs, which called competitive endogenous RNA (ceRNA). As the upstream and downstream of miRNA, RNAs constitute the relationship network between lncRNA, miRNA, and mRNA, which is very important for regulating RNA expression. In addition, lncRNAs play a role as a “molecular sponge,” directly or indirectly competitive binding with miRNA and finally weaken the effect of miRNAs on mRNAs [12–15].

Therefore, the establishment of survival-related ceRNA network of patients with ccRCC helps us to judge the close relationship between ceRNA network and the prognosis of patients. To understand the role of RNA network in tumorigenesis and find potential molecular therapeutic target to promote the prognosis of ccRCC. Compared with the general differentially expressed ceRNA network, the study of survival-related ceRNA network has a better application prospect in the prognosis of ccRCC.

## 2. Methods

### 2.1. Data Gathering and Sorting

RNA sequencing data and clinical data were gained from the GDC database (https://portal.gdc.cancer.gov/). TCGA (The Cancer Genome Atlas) is our database source. It collects clinical data and genomic variation and so on. TCGA is an important data source for cancer researchers. Our research follows the guiding principles of TCGA database. Because RNA sequencing data is gained from TCGA directly, the ethical permission is not required. We only selected RNA sequencing data of primary solid tumors for molecular analysis. The mRNA and lncRNA sequencing data included 537 primary ccRCC samples and 72 normal samples. The miRNA sequencing data included 516 primary ccRCC samples and 72 normal samples. Clinical information on the 537 patients is shown in Table 1.

### 2.2. Identification of Differentially Expressed RNAs

The differential expression lncRNAs (DElncRNAs), differential expression miRNAs (DEmiRNAs), and differential expression mRNAs (DEmRNAs) between the ccRCC and normal samples were analyzed using the edgeR package in the R 4.1.1 software. The cutoff value of differentially expressed RNAs (DERNAs) was ∣log2 fold − change (FC) | >2 and false discovery rate (FDR) < 0.01. The ggplot2 software package in the R software is used to visualize DERNAs.

### 2.3. Venn Diagram and Protein-Protein Interaction Network Construction

Venn diagram of DEmiRNA target genes intersected with DEmRNAs was analyzed by the Venn diagram package in the R 4.1.1 software. The protein-protein interaction data of DEmiRNAs or survival-related DEmiRNA target genes intersected with DEmRNAs were analyzed by STRING (http://string-db.org). PPI network was drawn by the Cytoscape software.

### 2.4. Survival Analysis

First, survival-related RNA was determined by univariate Cox regression analysis in the R software. Then, the survival-related RNA (*P* < 0.05) was selected for multivariate Cox regression analysis, and the RNA obtained from the results of multivariate Cox regression analysis was used to structure predictive survival models.

(1) $$\begin{array}{c} \left(\text{expressiongene}1\times b\text{ gene}1\right)+\left(\text{expressiongene}2\times b\text{ gene}2\right)+\cdots +\left(\text{expressiongenen}\times b\text{ genen}\right)=\text{Prognosis index }\left(\text{PI}\right). \end{array}$$

Patients were divided into two groups according to the median PI. Kaplan-Meier analysis was used to compare the survival and prognosis of the two groups. The receiver operating characteristic (ROC) curve for evaluating the predictive ability of the model was drawn by the R software.

### 2.5. Establishment of the ceRNA Network

The DERNAs and survival-related RNAs were used to structure ceRNA networks. The latent miRNA interactions between lncRNAs were selected according to the miRcode database primarily. Targeted mRNAs were predicted by using miRTarBase, miRDB, and TargetScan databases. Ultimately, the ceRNA network was established by the Cytoscape software. The website for obtaining data is as follows: http://www.mircode.org/, http://mirtarbase.cuhk.edu.cn/, http://www.mirdb.org/, and http://www.targetscan.org/.

### 2.6. Functional Enrichment Analysis

The mRNA in ceRNA network was enriched by Gene Ontology (GO) and Kyoto Encyclopedia of Genes and Genomes (KEGG) using KOBAS 3.0 (http://kobas.cbi.pku.edu.cn/kobas3/). The enrichment analysis was visualized by the R software.

### 2.7. Statistical Analysis

The rank sum test was used to analyze the relevance between clinical factors and RNA. The differences of survival curves were analyzed by log-rank test. The SPSS 24 statistical software was used for analysis. The GraphPad Prism 8, Cytoscape v3.8.2, and R 4.1.1 were used for drawing. There was statistical significance, *P* < 0.05.

## 3. Results

### 3.1. Visualization and Analysis of DElncRNAs, DEmiRNAs, and DEmRNAs

The RNA sequencing data of 537 patients with ccRCC was downloaded from TCGA database and screened out the DERNAs. The total 3,817 DERNAs were obtained; it includes 1,456 DElncRNAs (997 upregulated and 459 downregulated), 54 DEmiRNAs (33 upregulated and 21 downregulated), and 2,307 DEmRNAs (1,546 upregulated and 761 downregulated). Ultimately, we visualized these DERNAs by heat map and volcano maps in Figure 1. Venn diagram of DEmiRNA target genes intersected with DEmRNA. We intersect 2,307 DEmRNAs with 331 DEmiRNA target genes. 17 intersecting mRNAs were obtained for subsequent ceRNA and PPI network construction. We also established a PPI network with DEmiRNA target genes. The results are shown in Venn diagram (Figure 2(a)). PPI networks were constructed by STRING (Figures 2(b) and 2(c)).

### 3.2. Visualization and Analysis of Survival-Related RNAs in ccRCC

The correlation between survival status and DERNAs was evaluated by univariate Cox regression analysis. RNAs with *P* value less than 0.05 were survival-related RNAs, the total 42 survival-related DERNAs (6 mRNAs, 32 lncRNAs, and 4 miRNAs) were obtained. The top 6 survival-related mRNAs, 15 lncRNAs, and 4 miRNAs are shown in Figure 3.

### 3.3. Establishment of Predictive Survival Models

The RNA with *P* < 0.05 was selected by univariate Cox regression analysis, which was considered to be closely related to survival, and then, multivariate Cox regression analysis was used for these strongly correlated RNAs. Finally, a total of nine lncRNAs (COL18A1-AS1, FGF12-AS2, LINC00443, AC009093.1, WT1-AS, TRIM36-IT1, AC110619.1, TCL6, HOTTIP), two miRNAs (mir-155 and mir-21), and three mRNAs (PRELID2, COL4A4, ERMP1) were identified. Then, we use the above results to establish a predictive survival model.

(2) $$\begin{array}{c} \left(-0.16658\times \text{FGF}12-\text{AS}2\text{ expression}\right)+\left(0.08625\times \text{WT}1-\text{AS expression}\right)+\left(-0.1609\times \text{COL}18\text{A}1-\text{AS}1\text{ expression}\right)+\left(0.11859\times \text{AC}009093.1\text{ expression}\right)+\left(0.12695\times \text{TRIM}36-\text{IT}1\text{ expression}\right)+\left(-0.29689\times \text{LINC}00443\text{ expression}\right)+\left(-0.09373\times \text{TCL}6\text{ expression}\right)+\left(0.08703\times \text{HOTTIP expression}\right)+\left(0.09382\times \text{AC}110619.1\text{ expression}\right)=\text{PIlncRNA}.\left(0.13856\times \text{mir}-155\text{ expression}\right)+\left(0.52054\times \text{mir}-21\text{ expression}\right)=\text{PImiRNA}.\left(-0.29343\times \text{PRELID}2\text{ expression}\right)+\left(-0.34645\times \text{ERMP}1\text{ expression}\right)+\left(-0.21887\times \text{COL}4\text{A}4\text{ expression}\right)=\text{PImRNA}. \end{array}$$

According to the PI value of each patient, they were divided into high or low risk groups. We found that, based on K-M analysis, among the three groups of RNAs, the survival rate was higher in the low-risk group (Figures 4(a)–4(c)). The survival model to predict 3-year survival was assessed by drawing the ROC curve. The areas under the curves (AUCs) of PIlncRNA, PImiRNA, and PImRNA were 0.717, 0.643, and 0.666 (Figures 4(d)–4(f)). The results indicated that the survival models of ceRNA perform very well in predicting the clinical prognosis of ccRCC. The survival status, RNA expression profile, and risk score are shown in Figure 5. The relevance of these RNAs with other clinical features was evaluated by rank sum test. Clinical features consist of age (<46/≥46), tumor stage (I-II/III-IV), gender (male/female), and race (white/nonwhite). The results also indicated that RNA in the survival model was correlated with tumor stage significantly which is shown in Figure 6. These survival-related RNAs can be used as potential therapeutic indicators to evaluate the tumor progression of ccRCC. Then, we determined the relevance between OS. Multivariate Cox regression analysis and clinical features showed that risk level and tumor stage affected tumor prognosis directly (Table 2).

### 3.4. Construction of a Differentially Expressed ceRNA Network in ccRCC

In view of the differentially expressed RNAs, these included 17 pairs of miRNA-mRNAs and 161 pairs of lncRNA-miRNA. The ceRNA network included 17 DEmRNAs, 81 DElncRNAs, and 9 DEmiRNAs which were constructed as follows (Figure 7(a)).

### 3.5. Construction of a Survival-Related ceRNA Network in ccRCC

In view of the survival-related DERNAs, these included 12 pairs of miRNA-mRNAs and 4 pairs of lncRNA-miRNA. The ceRNA network included 12 DEmRNAs, 4 DElncRNAs, and 2 DEmiRNAs which were constructed as follow (Figure 7(b)). By comparing the differences between the two networks, we found that the ceRNA network based on survival model is more clearly and easier to find the direct relationship between lncRNA-miRNA-mRNA.

### 3.6. Enrichment Analysis by GO and KEGG Pathway

Subsequently, we investigated the downstream pathway of mRNAs in the ceRNA network. GO and KEGG functional enrichment analyses were carried out, including molecular functions, cellular components, and biological processes from the GO analysis and pathways from KEGG. The biological processes were mainly enriched in “cytokine-mediated signaling pathway,” the molecular function was mainly enriched in “extracellular matrix structural constituent,” and the cellular components were enriched in “phagocytic vesicle.” The KEGG analysis suggested that the “ECM-receptor interaction,” “Pathways in cancer,” and “Chemokine signaling pathway” were the main pathways (Figure 8).

## 4. Discussion

Renal cancer is a progressive malignant tumor with high morbidity and mortality rate. Clear cell renal carcinoma accounts for 70-80% of all renal cell carcinoma [16]. It is the most representative subtype. From a point of view, with the gradual deepening of our understanding of the molecular and genetic mechanisms of ccRCC, we have made progress in the prevention, diagnosis, and treatment of this cancer. However, ccRCC is still the main cause of cancer-related death. Most studies of ccRCC focus on identifying the abnormal mechanism of a single cause. However, the mechanism of cancer occurrence and development is complex and changeable. It is hard to see the whole picture only by studying a single gene. Therefore, studying the network regulatory interaction between all RNA encoded by the genome, especially noncoding RNA and coding RNA, which is helpful to find specific biomarkers for patients with ccRCC.

The RNA transcriptome of cancer is significantly different from that of normal samples, so most researchers also believe that the ceRNA spectrum in cancer may be different from that in normal state, and more and more evidences show that the abundance and activity of ceRNA will be deregulated or reprogrammed in cancer. The cross-talk of ceRNA is a posttranscriptional regulation, which is centered on miRNA and connects coding RNA and noncoding RNA [17]. A recent study found that the expression of lncRNA LINC01133 decreased in gastric cancer tissues and gastric cancer cell lines, and its low expression was positively correlated with the progression and metastasis of gastric cancer. Through bioinformatics analysis and luciferase reporter gene analysis, this study identified miR-106a-3p as the direct target of LINC01133, indicating that LINC01133, as the ceRNA of miR-106a-3p, plays a role in the progression of gastric cancer [18]. Furthermore, previous study showed that long noncoding RNA (lncRNA) XLOC006390 may be used as ceRNA to competitively bind miR-331-3p and miR-338-3p, then downregulate the expression of its target genes, so as to promote the occurrence and metastasis of cervical cancer [19]. The high expression of lncRNA-CDC6 in breast cancer tissues is positively correlated with the clinical stage of breast cancer. In addition, lncRNA-CDC6 promotes the progression and metastasis of breast cancer through direct competitive combination of microRNA-215 (miR-215) as competitive endogenous RNA (ceRNA), which provides a new biomarker for clinical prognosis of breast cancer [20]. MicroRNA-206 affects the prognosis of ccRCC by targeting ZEB2 [11]. This finding is also consistent with the conclusions in this study.

We found a recent study focused on ceRNA network on ccRCC patient. Gong et al. found that the established ceRNA network was closely related in the progression and metastasis of ccRCC and 3 lncRNAs that may be related to ccRCC prognosis [21]. However, the difference or advantage of our study lies in a more accurate survival-related ceRNA network [22, 23]. Among DERNAs, the total 2,307 DEmRNAs (761 downregulated and 1,546 upregulated), 54 DEmiRNAs (21 downregulated and 33 upregulated), and 1,456 DElncRNAs (459 downregulated and 997 upregulated) were screened. Then, we conducted a univariate Cox regression analysis between DERNAs and clinical factors, selected RNA with *P* less than 0.001 for multivariate Cox regression analysis, and constructed a survival-related ceRNA network included 9 lncRNAs, 2 miRNAs, and 3 mRNAs, which are the key RNAs to achieve molecular functions. We think our research may be more accurate, representative, and more suitable for future clinical applications.

Our study still had several limitations. Such as the AUC value of our model was 0.717, 0.643, and 0.666. The values of the latter two groups are less than 0.7, but very close, which may be due to the smaller selection range (∣log2 fold − change (FC) | >2 and false discovery rate (FDR) < 0.01) and more accurate DERNAs, resulting in the AUC value less than 0.7.

## 5. Conclusions

In summary, we established a predictive survival model based on multivariate Cox regression analysis, which has great prospect in future clinical application and becomes a potential target to judge the prognosis of patients. We screened high-risk patients and strengthened personalized treatment through sequencing results which are hope to promote the long-term prognosis for ccRCC patients. Meanwhile, we firstly constructed an lncRNA-miRNA-mRNA regulatory ceRNA network and then constructed a ceRNA network based on survival model, which is different from the same type of research. The establishment of ceRNA network provides therapeutic targets and new potential prognostic indicators for predicting ccRCC patients' prognosis and reduces the selection range of therapeutic targets through survival analysis.

## Figures and Tables

**Figure 1:** Differential expression of lncRNAs, miRNAs, and mRNAs. (a) Volcano plot and (b) heat map of DElncRNAs. (c) Volcano plot and (d) heat map of DEmiRNAs. (e) Volcano plot and (f) heat map of DEmRNAs. The red point in the volcano plot represents upregulated RNAs, and green point represents downregulated RNAs.

**Figure 2:** Venn diagram and PPI network of DEmiRNA target genes intersected with DEmRNAs. (a) Venn diagram: target genes of DEmiRNAs intersected with DEmRNAs. (b) PPI network: target genes of DEmiRNAs by Cytoscape. The degree decreased from inside to outside, and the color changed from dark to light. (c) PPI network: 17 intersected mRNAs between 2,307 DEmRNAs and 331 DEmiRNA target genes. The degree decreased from inside to outside, and the color changed from dark to light.

**Figure 3:** Forest plots of the hazard ratios (HR) of the survival-related RNAs in ccRCC. (a) HR of top 15 survival-related lncRNAs. (b) HR of 4 survival-related miRNAs. (c) HR of 6 survival-related mRNAs. HR < 1 indicated the low risk RNAs, and HR > 1 indicated the high risk RNAs.

**Figure 4:** Kaplan-Meier (K-M) curves and ROC curves for PI in ccRCC patients. (a) lncRNA model: K-M survival curves between high-risk and low-risk groups. (b) miRNA model: K-M survival curves between high-risk and low-risk groups. (c) mRNA model: K-M survival curves between high-risk and low-risk groups. (d) Time-dependent ROC curve analysis for survival prediction by PIlncRNA. (e) Time-dependent ROC curve analysis for survival prediction by PImiRNA. (f) Time-dependent ROC curve analysis for survival prediction by PImRNA.

**Figure 5:** The patients were divided into low-risk group and high-risk group and then conduct prognostic classifier analyses. (a) Risk score distribution based on lncRNA. (b) Risk score distribution based on miRNA. (c) Risk score distribution based on mRNA. (d) Survival status based on lncRNA in two groups. (e) Survival status based on miRNA in two groups. (f) Survival status based on mRNA in two groups. (g) lncRNA heat map in two groups. (h) miRNA heat map in two groups. (i) mRNA heat map in two groups.

**Figure 6:** Clinical factors of RNAs related to prognosis of ccRCC. The brighter the color of each cell, the smaller the *P* value. The number in the cell is the *P* value.

**Figure 7:** (a) The differential expression lncRNA-miRNA-mRNA competing endogenous RNA network. (b) Survival-related ceRNA network in ccRCC. The red indicated upregulated RNAs, and the blue indicated downregulated RNAs. The ellipse indicated mRNAs. The diamond indicated lncRNAs, and the round rectangle indicated miRNAs.

**Figure 8:** GO and KEGG pathway enrichment analyses of genes in the lncRNA-miRNA-mRNA competing endogenous RNA network. (a) Biological process. (b) Cellular component. (c) Molecular function. (d) KEGG pathways.

**Table 1:** Corresponding clinical features of 537 patients with clear cell renal cell carcinoma.

Items	Patients, *N* = 537	
	*N*	%
Age		
<46	61	11.3594
≥46	476	88.6406
Gender		
Male	346	64.4302
Female	191	35.5678
Race		
White	466	86.7784
Nonwhite	71	13.2216
Tumor stage		
Stage I/II	329	61.2663
Stage III/IV	208	38.7337
Survival status		
Alive	375	69.8324
Dead	162	30.1676

**Table 2:** Univariate and multivariate Cox regression analysis of overall survival.

Overall survival	Univariate Cox analysis			Multivariate Cox analysis		
	HR	95% CI	*P* value	HR	95% CI	*P* value
Age (<46/≥ 46)	2.263268094	1.1553-4.4337	0.017273078			
Gender (male/female)	1.057248789	0.7681-1.4552	0.732716575			
Race (white/nonwhite)	0.734643916	0.3868-1.3952	0.346052689			
Tumor stage (I-II/III-IV)	4.156665354	2.9807-5.7965	4.57*E*-17			
lncRNA cohort				3.033	2.139-4.300	4.70*E*-10
miRNA cohort				3.525	2.496-4.978	8.41*E*-13
mRNA cohort				3.49	2.470-4.931	1.39*E*-12
lncRNA signature (low risk group/high risk group)	3.985610434	2.7434-5.7903	4.00*E*-13	2.74	1.857-4.043	3.85*E*-07
miRNA signature (low risk group/high risk group)	2.006770711	1.4465-2.784	3.05*E*-05	1.571	1.126-2.194	0.00793
mRNA signature (low risk group/high risk group)	2.775537016	1.9666-3.9171	6.34*E*-09	1.595	1.141-2.228	0.00626

## Data Availability

All the RNA sequencing data that used in present study were deposited in TCGA database.
